# The crescendo pulse frequency of shear stress stimulates the endothelialization of bone marrow mesenchymal stem cells on the luminal surface of decellularized scaffold in the bioreactor

**DOI:** 10.1080/21655979.2022.2039502

**Published:** 2022-03-31

**Authors:** Yuhao Jiao, Yuanguo Zhang, Yonghao Xiao, Yuehao Xing, Zhiwen Cai, Cong Wang, Zhengtong Zhou, Zengguo Feng, Yongquan Gu

**Affiliations:** a Department of Vascular Surgery, Xuanwu Hospital, Capital Medical University, Beijing, China; b School of Materials Science and Engineering, Beijing Institute of Technology, Beijing, China

**Keywords:** Vascular tissue engineering, biomechanical stimulation, frequency, shear stress, endothelial cell (EC), bone mesenchymal stem cells (MSC)

## Abstract

A completely confluent endothelial cell (EC) monolayer is required to maintain proper vascular function in small diameter tissue-engineered vascular graft (TEVG). However, the most effective method for EC attachment to the luminal surface and formation of an entire endothelium layer that works in vitro remains a complicated challenge that requires urgent resolution. Although pulsatile flow has been shown to be better suited for the generation of functional endothelium, the optimal frequency setting is unknown. Several pulsatile flow frequencies were used to implant rat bone mesenchymal stem cells (MSC) into the lumen of decellularized porcine carotid arteries. The endothelium's integrity and cell activity were investigated in order to determine the best pulse frequency settings. The results showed that MSC were maximally preserved and exhibited maximal morphological changes with improved endothelialization performance in response to increased pulse stimulation frequency. Increased pulse frequency stimulation stimulates the expression of mechanoreceptor markers, cytoskeleton reorganization in the direction of blood flow, denser skeletal proteins fibronectin, and stronger intercellular connections when compared to constant pulse frequency stimulation. MSC eventually develops an intact endothelial layer with anti-thrombotic properties on the inner wall of the decellularized tubular lumen. Conclusion: The decellularized vessels retain the three-dimensional structure of the vasculature, have a surface topography suitable for MSC growth, and have good mechanical properties. By increasing the frequency of pulsed stimulation, MSC endothelialize the lumen of the decellularized vasculature. It is expected to have anti-thrombotic and anti-neointimal hyperplasia properties after implantation, ultimately improving the patency of TEVG.

## Highlights

- Pulsed stimulation promotes MSC proliferation and differentiation on the inner surface of decellularized blood vessels.
- Maximum cell retention was achieved with increasing frequency of pulse stimulation
- Pulse stimulation promoted MSC differentiation to endothelial cells, forming an intact and functional endothelial layer.

## 1. Introduction

Cardiovascular and cerebrovascular illness are the main causes of mortality and morbidity globally. As the population ages and risk factors grow, there is a significant therapeutic need for TEVG[1]. The primary complications associated with small diameter TEVG (<6 mm) are thrombosis and neointimal hyperplasia, which result in poor long-term patency. These complications are primarily caused by the vascular graft lacking a confluent and functional endothelial layer capable of performing biological functions following implantation [2].

It is widely established that vascular EC development occurs in three distinct ways after *ex vivo* transplantation: transanastomotic migration, transmural infiltration, and fallout healing [3]. The strategy for cell-free *in situ* tissue engineering is to accomplish *in situ* endothelialization by physically and chemically modifying the luminal surface of the vascular graft in order to attract EC and endothelial progenitor cells [4]. However, for long segments of vascular grafts, it is not easy to achieve complete endothelialisation in the short term [5]. Thrombotic occlusion is caused by the lack of a functional endothelium on small-diameter vascular grafts [6]. Stimulation by transmural interstitial flow eventually leads to occlusion due to neointimal hyperplasic [7].

Natural arteries are not merely tubes for blood transfer, they are constantly exposed to the pulsatile blood flow waves generated by the heart’s systolic and diastolic movements. ECs are primarily exposed to shear stress and circumferential stretch derived by blood flow, which convert mechanical stimulation to intracellular signals that affect cellular function, promoting EC adhesion, proliferation, migration, permeability, remodeling and regulating gene expression [8,9]. Endothelialization of small diameter TEVG *in vitro* has been one of the most promising strategies for increasing anti-thrombotic activity, inhibiting intimal hyperplasia and increasing patency rates. However, the critical challenge is EC washing and shedding upon implantation when subjected to genuine blood flow pulses *in vivo*. The largest problem becomes pretreatment *in vitro* to allow them to withstand physiological levels of shear stress[10].

Cell retention and normal function of the endothelium is an even more daunting task to generate functional endothelium. EC are subjected to a broad variety of mechanical stimulation, and their sensitivity adapts in response to particular variances in flow patterns, such as the amplitude, direction, temporal gradients and frequency content [11]. Xanthis and colleagues demonstrated that β1 integrin is the crucial sensor of force direction by using in vitro flow systems and magnetic tweezers. Unidirectional flow normalizes the EC and maintains vascular homeostasis [12]. According to Gong and coworkers, EC exhibit superior cell retention, the formation of denser and regular F-actin microfilament bundles in the same direction, the assembly of thicker and highly crosslinked fibronectin, and a significant inhibition of cell apoptosis when subjected to physiological pulsatile flow [13]. Liu *et al* have demonstrated that gradually increasing shear stress with appropriate time-steps and amplification could improve EC retention, yielding a complete endothelial-like monolayer both *in vitro* and *in vivo*, the modest increase group with slight amplification (10% increase/h) demonstrated a significant improvement in cell retention, allow additional time for ECs to gradually acclimatize to the changing of environment [14]. Our research group also confirmed this conclusion that stepwise increased shear stress could enhance retention rate, strengthen cell–cell and cell–extracellular matrix connections [15]. The vast majority of studies made on vascular constructs have limited their culture conditions to constant parameters, mostly strain amplitude and time dependency (stretch time, relaxation time, frequency) [16].The optimal pulse frequency *in vitro* is still uncertain.

The present study sought to investigate the optimal pulse frequency to achieve maximum cell retention, to achieve maximum morphological changes and EC function. Four groups of different frequencies were set up to perform pulsed shear stress stimulation on cells implanted into the inner surface of decellularized vessels of porcine carotid arteries at the same time step, and EC marker expression, cytoskeleton and function were investigated on the surface of the tubular scaffold to explore the optimal pulse frequency.

## 2. Materials and methods

### 2.1 Preparation of decellularized vascular matrix

The decellularized porcine carotid artery scaffolds were prepared as described in our previous study [17,18]. Briefly, Carotid arteries from porcine (internal diameter 3 mm, length 5 cm) were obtained, the lumen was flushed with heparin saline to remove blood clots, the outer membrane and fatty tissue were stripped, the vessels were washed with phosphate buffered saline (PBS) for one day, the vessels were shocked in 1% Triton X-100 solution (Labest Biological Technology, Beijing, China) for 24 hours (100 r/min), shocked with 0.3% sodium dodecyl sulfate (SDS, Hanran Biological Technology, Shanghai, China) for 72 hours and changed daily. Decellularised vessels were washed with PBS solution to remove residual detergent. The decellularised vessels were finally cross-linked using N-(3-dimethylaminopropyl)-N0ethylcarbodiimide hydrochloride (EDC) and N-hydroxysuccinimide (NHS) to enhance mechanical properties and immobilize heparin sodium (Beijing Solarbio Science & Technology, China). The vessels were finally dispensed and disinfected using Y-rays.

### 2.2 Cell culture

MSC were isolated from 3–4 week old Sprague-Dawley male rat as previously described [19].Briefly, Rats were anesthetized, neck pulled and disinfected by immersion in 75% alcohol, the femur was taken, washed three times with PBS, the bone marrow cavity was rinsed with Dulbecco’s Modified Eagle Medium (DMEM, Gibco, USA), the bone marrow was isolated with lymphocyte isolation solution Ficoll (Sigma, USA), and the complete medium DMEM, supplemented with 10% fetal bovine serum(FBS, Gibco, USA), 100 U/ml penicillin, 100 mg/ml streptomycin, 50 ng/ml vascular endothelial growth factor (VEGF, Invitrogen USA) and 50 m/ml heparin (gibco, USA). The cells were placed in static culture inside the cell culture plastic, and when the cells were fused to 80%, they were passaged, using 3–5 generations of cells. Flow cytometry was used to identify the cells.

### 2.3 Cell growing and dynamic culture in bioreactor

The process of dynamic cultivation is shown in Figure 1. MSC fused to 80% in the cultureplastic was digested using trypsin-EDTA (Gibco, USA). The cells suspension (1*10^6 cell/scaffold) was gently pipetted into the lumen of the scaffold tube (Figure 1 A), with the ends fixed in the rotating chamber (Figure 1B). The luminal circuit connectors of the rotatory chamber are threaded swivel connectors to permit the rotation of the chamber without twisting of the tubes. Install the peristaltic pumping system inside the EBER TEB500 bioreactor (Figure 1C), consisting of the reservoir bottle, connecting lines and the closed loop of the culture chamber. Close the TEB500 door to create a sterile environment inside. The bioreactor was connected to an external computer and controlled by using the software provided by the manufacturer, with the temperature set at 37°C, 5% CO2, 10% O_2_; the control motor speed and peristaltic pumping speed and frequency were controlled by changing the software variables. [Figure 1D]. The motor was started at a constant speed of 6 rotation/h to facilitate cell settlement and adhesion within the artificial vessel to promote the uniform distribution of cells within the lumen of the stent tube [15].

The shear stress generated by the bioreactor was increased step by step from 0.1 ml/min every 30min, according to the equation for shear stress in blood vessels Q = τωh2/ 6μ, where Q is the volumetric flow rate, τ is the average shear stress of MSC exposure, and μ is the dynamic viscosity of the culture medium. in this study was 0.7600 cp, It is well known that the average shear stress of ECs in arteries within the range of 10–70 dyn/cm [2], in order to promote MSC differentiation to arterial ECs, All reached 34 ml/min (12.9 dyn/cm2) after seven days. The frequency was different in the four groups, group A was the static culture group with medium change every two days group; group B was the constant 60s pulse, group C was the constant 1 s pulse, and group D was the gradually increased the pulse frequency, increasing the frequency by 10s per day. The vessels were removed after seven days of culture to investigate the vessels and cells. All connecting tubes were sterilized by high temperature and autoclaving.

**Figure 1.,:** The decellularized vessels are secured in the culture chamber by knots at both ends and can be rotated at a uniform speed by a digitally driven rotating device, with a peristaltic pump system providing shear stress to the surface MSC.

Figure 1A. The digested cell suspension is planted onto the inner surface of the decellularized vessel lumen.Figure 1B. Decellularized vascular surgical sutures are knotted and secured to a matching interface under aseptic conditions on an ultra-quiet table and installed into the rotating culture chamber. Figure 1C. The ends of the rotating culture chamber were connected to a circuit filled with culture medium at 6 r/h for 4 hours to achieve uniform coverage of cells in the tubular structure.Figure 1D Start the peristaltic pump system and incubate statically for the first 48 hours and then gradually increase the flow rate by 0.1 ml/min every 30 min.

### 2.4 Cell viability evaluation

To assess the effect on MSC under pulsed stimulation at different frequencies, different groups of cells growing on the surface of decellularised vessels were stained using Calcein/PI Cell Viability Assay Kit (Beyotime, China) to assess cell viability and death. Calcein AM is a cell-permeant dye that can be used to determine cell viability. In live cells the nonfluorescent calcein AM is converted to a green-fluorescent calcein, after acetoxymethyl ester hydrolysis by intracellular esterases. Since dead cells lack esterase or have deficient esterase activity, they are unable or rarely able to produce calcein and therefore only live cells are stained with intense green fluorescence. The red-fluorescent nucleic acid dye Propidium Iodide (PI) cannot penetrate the cell membrane of living cells and can only stain dead cells where the integrity of the cell membrane has been disrupted. Cells on the lumenal surface of the tubes were observed with an inverted fluorescence microscope (TCS SP5; Leica, Germany). Three fields of view (magnification: 400×, area: 0.25 mm2) were randomly selected, and the cell count was determined using Image J Pro software.

### 2.5 Scanning electron microscopy observation (SEM)

After seven-day cultivation under shear stress in the bioreactor, the vessels were fixed with 2.5% glutaraldehyde (Beijing Solarbio Science & Technology, China) overnight at 4°C, and dehydrated in a series of graded ethanol (25%, 50%, 75%, 95% and 100%) before lyophilization. Dissect the vessel with scissors to expose the inner surface of the lumen. The freeze-dried samples were then mounted onto stubs, sputtered with platinum, and observed with a scanning electron microscope (SEM. SU8010, Hitachi, Japan)

### 2.6 HE staining

Decellularised vessels were removed after seven days of culture, washed three times with PBS, fixed using 4% paraformaldehyde for 24 hours, dehydrated in graded xylene and graded ethanol, embedded in paraffin and cut into 5um serial sections and stained using hematoxylin and eosin to assess the luminal cells. Three fields of view (magnification: 400×, area: 0.25 mm2) were randomly selected,,microscopic examination using a microscope (IX71, Olympus, Japan)

### 2.7 Immunofluorescence (IF)

Differences in EC-specific protein expression levels between the different groups were determined by immunofluorescence. The samples from each experimental group were fixed in 4% paraformaldehyde at room temperature for 15 minutes. Samples were washed three times for five minutes each with PBS, permeabilizing with 0.5% Triton-X-100 solution (Sigma, St. Louis, MO, USA) and blocking with 1% donkey serum albumin (Sigma, St. Louis, MO, USA) to avoid nonspecific staining, the sections were stained with the following rabbit anti-rat antibodies (1:100): anti-CD31, (PA5-32,321, Thermo Fisher scientific, USA), anti-VEGFR2 (26,415-1-AP, Proteintech, China), anti-VE-cadherin(36–1900, thermo Fisher scientific, USA), anti-F-actin(FITC Phalloidin, CA1620-300 T, Solarbio, China), anti-Fibronectin(PA5-29,578, thermo Fisher scientific, USA, anti-vinculin(26,520-1-AP, Proteintech, China),anti-Thrombomodulin(14,318-1-AP, Proteintech, China) at 4°C overnight. After the complete rinses with PBS, the samples were incubated with the 488-conjugated donkey anti-Rabbit IgG and donkey anti-Mouse (Invitrogen, Carlsbad, CA,USA) at 37°C for 2 h, and followed by staining with DAPI(D1306, thermo Fisher scientific, USA).The samples were observed under confocal microscopy. Three randomly selected fields of view were used to measure the immunofluorescence intensity using Image-Pro software.

### 2.8 Gene expression by real-time RT-PCR analysis

To compare the mRNA expression levels of EC-tagged genes at different frequencies between groups, the cultured vessels were stored in liquid nitrogen and total RNA was extracted using RNA Extraction Liquid Molecular Biology Reagent (G3013, Servicebio, Wuhan, China) according to the manufacturer’s instructions. Total RNA was extracted using the RNA Extraction Liquid Molecular Biology Reagent (G3013, Servicebio, Wuhan, China) according to the manufacturer’s instructions, taking OD at 260 nm and 280 nm to determine sample concentration and purity. Reverse transcription was performed using the SweScript RT I First Strand cDNA Synthesis Kit (G3330, Seervicebio, Wuhan, China) for reverse transcription. Real-time PCR was performed using a fluorescent quantitative PCR instrument (ABI, S tepe).The relative mRNA expression levels for CD31, VEGFR2 (flk-1) were estimated and normalized to β-actin.Each sample was tested in triplicate.

### 2.9 Statistical analysis

All data are presented as mean ± standard deviation (SD). Statistical analysis was performed using one-way analysis of variance (ANOVA) for multiple comparisons by Graph Pad Prism. P < 0.05 was considered statistically significant.

## 3.Results

In order to investigate the optimal pulse frequency for MSC to form an intact and functional endothelial layer on the inner surface of decellularized vessels, four different frequencies of pulsed shear stress were set up in this experiment. Live and dead cells were used to identify the effects on cells at different frequencies. The luminal surface morphology and cell coverage were observed using electron microscopy, the distribution of cells in the vessels was determined using HE staining, and the expression of endothelial cell mechanoreceptors, cytoskeleton and functional proteins in MSC was determined by immunofluorescence.

### 3.1. Cell viability and morphology

After seven days of incubation, MSCs in the static culture group showed a disordered arrangement with variable cell morphology and more dead cells (Figure 2a), while the constant 60S frequency group showed deformation of cells with *consistent* directional effect and less number of dead cells than static culture group (Figure 2b). 1S group showed a large number of dead cells (Figure 2c). A more pronounced cytoskeletal rearrangement, parallel to the direction of flow, was seen in the pulsed group with gradually increasing frequency; only a few dead cells are visible (Figure 2d). Cell counts suggested that the static culture group and the 1S frequency group had a higher proportion of dead cells, while the constant 60S and gradually increasing frequency groups had a relatively smaller proportion of dead cells. (Figure 2e).

**Figure 2.** Staining for live and dead cells on the luminal surface of the tubes. static(a); constant 60s pulse(b), constant 1 s pulse(c), gradually increased the pulse frequency (d). live and dead cell counts in different groups (e). scale bars = 100 um.

### 3.2 Scanning electron microscopy observation

After seven days of culture, the inner surface of the tube lumen was observed using electron microscopy scanning and it was seen that the static culture group formed a smooth basement membrane layer on the inner standard surface and no obvious cell morphology was seen (Figure 3a). The constant 60S group could be seen to have a cobblestone-like appearance with some directionality (Figure 3b). In the constant 1S group, the basement membrane could be intercalated, but there was a large gap between the cells, and only some residual cells remained (Figure 3c). A cobblestone-like arrangement in the direction of blood flow was evident in the gradually increasing frequency group (Figure 3d).

**Figure 3.** Scanning electron microscopy of the inner surface of the tube lumen. static(a); constant 60s pulse(b), constant 1 s pulse(c), and gradually increased the pulse frequency (d).

### 3.3 HE

HE staining of vascular ring sections showed that no obvious cellular components remained in any of the four groups of decellularized vessels, and the preserved intact elastic lamina layer was visible under the tunica intima. In the static culture group, cells grew densely, stacked in multiple layers and irregularly arranged (Figure 4a). After dynamic culture, a smooth monolayer of an endothelial layer was seen to form on the luminal surface of the tubes (Figure 4b). In the gradually increasing frequency group, a thicker basement membrane was seen and the cells were more closely arranged (Figure 4d). While in the 1S frequency group the cells were loosely distributed and failed to maintain a continuous smooth endothelial layer (Figure 4c).

**Figure 4.** H&E staining static(a); constant 60s pulse(b); constant 1 s pulse(c); gradually increased the pulse frequency (d). scale bars = 100 um.

### 3.4 Immunofluorescence expression of endothelial cell mechanoreceptors

Immunofluorescence staining of cells on the luminal surface of the tubes showed that MSC did not express any of the three mechanoreceptor proteins in the static culture group without shear stress stimulation (Figure 5a, E, I). 60S constant shear stress showed fluorescence expression around the nucleus (Figure B, F, J), Gradually increasing frequency groups showed a neater and more complete arrangement of cells, with immunofluorescent proteins distributed around the oval-shaped nuclei, parallel to the direction of blood flow(Figure D, H, L).and 1S group could be interspersed with scattered cell expression.(C, G, K) Quantitative fluorescence analysis showed a significant increase in the expression of the three mechanoreceptor proteins in the experimental group compared to the first three groups (P < 0.001). (Figure 5 M, N, O)

**Figure 5.** Immunofluorescent staining for EC-specific proteins CD31, VE-cadherin and VEGFR2 (flk-1). static group (A, E, I). constant 60s (B, F, J);constant 1 s pulse(C, G, K); gradually increased the pulse frequency (D, H, L). immunofluorescence staining for CD31 (m), VE-cadherin (n) and VEGFR2 (o) was quantified using imagej by the meaning of fluorescence intensity. *P < 0.05, **P < 0.01, ***P < 0.001. scale bars = 50 um.

### 3.5 Immunofluorescence expression of F-actin and fibronectin

Figure 6 shows F-actin and Fibronectin in MSC on the inner surface of the decellularized tubular lumen after seven days of culture. Staining for cytoskeleton and Fibronectin was seen in the static culture group as disordered, disorganized microfilaments, The dense nuclei are surrounded by only a sparse, thinly layered, scattered fibrin network. (Figure 6a, e). After shear stress, the 60S group was seen to have significantly more microfilaments and appeared around the nucleus, lined up in the direction of blood flow. (Figure 6 B F).1S group saw larger defective areas in the selected region with significantly less cell coverage than before. Thicker F-actin and denser Fibronectin were seen in the experimental group, the fibers are intertwined and cross-linked into a dense network that covers the surface of the lumen.(Figure 6 D, H). Fluorescence intensity quantification showed a statistically significant difference in the experimental group compared to the first three groups.

**Figure 6.** Immunofluorescent staining of F-actin and fiibronectin. static group (a, e). constant 60s (b, f);constant 1 s pulse(c, g); gradually increased the pulse frequency (D, H,). immunofluorescence staining for F-actin (i), fibronectin (j) was quantified using image J pro by the meaning of fluorescence intensity. *P < 0.05, **P < 0.01, ***P < 0.001. scale bars = 100 um.

### 3.6 Immunofluorescence of functional protein expression in endothelial cells

Thrombomodulin, also known as CD141, is an endothelial cell surface glycoprotein that forms a 1:1 complex with the coagulation factor thrombin and plays an essential role as a natural anticoagulant. Vinculin is necessary to form junctional fingers, which are important connecting structures in the budding of angiogenesis, which are formed transiently under increased pressure, thus maintaining the integrity of the blood vessels. No functional expression of endothelial cells was observed in static culture alone (Figure 7a,e), and after hemodynamic stimulation, all dynamic culture groups expressed antithrombotic and vinculin proteins, Compared to the constant frequency group, there was a significant difference in immunofluorescence intensity for pulses of gradually increasing frequency (Figure 7i,j)

**Figure 7.** Immunofluorescent staining of thrombomodulin and vinculin. Static group (a, e). constant 60s (b, f);constant 1 s pulse(c, g); gradually increased the pulse frequency (D, H,). Immunofluorescence staining for Thrombomodulin (i), Vinculin (j) was quantified using Image J pro by the meaning of fluorescence intensity. *P < 0.05, **P < 0.01, ***P < 0.001. Scale bars = 100um.

### 3.7 Gene expression of EC-specific markers

In order to compare the degree of differentiation of MSC to EC-like cells under different frequencies of pulse stimulation, the mRNA expression levels of the mechanoreceptors of EC, i.e. CD31 and VEGFR2, were analyzed by real-time PCR, respectively. As shown in Figure 8, the marker genes of CD31 and VEGFR2 were significantly upregulated after dynamic culture compared with static culture, and the pulse group with gradually increasing frequency was significantly higher than the constant frequency group, which was consistent with the fluorescence quantification results.

**Figure 8.** RT-PCR analysis for the EC marker genes expressions. data are expressed as mean ± SD. *P < 0.05, **P < 0.01, ***P < 0.001.

## 4. Discussion

Research related to TEVG has been performed for several decades, investigators have focused on constructing vascular grafts with mechanical properties and biological functions similar to those of native vessels [20,21]. While *in vitro* tissue engineering is difficult to form a complete endothelial layer and mature elastic fibers in a short period of time [22]. Extracellular matrix (ECM) scaffolds preserve the three-dimensional architecture and the two most vital proteins collagen and elastin, which elastin is to confer compliance and collagen is responsible for the resistance to rupture [23]. Our previous experiments found that decellularized vessels after chemical cross-linking arrangement with mechanical properties matching those of the autologous vasculature. Besides, the substrate stiffness, spatial patterning and basement membrane accelerating cells adherence to artificial surfaces.The superior biocompatibility provides beneficial bioactive components for stem cell differentiation, thus accelerate expediting endothelialization [24].

Multiple studies have confirmed that endothelial cells can only tolerate the shear stress of 5 dyn/cm [2] due to the limited proliferation capacity and rapid cell function attenuation [25,26]. Bone-MSC have unique characteristics and properties, higher proliferative potential and lower immunogenicity and immunoregulatory properties; the above features suggest that MSC are ideal seed cells for vascular tissue engineering [27].

The biggest problem facing small diameter TEVG is the formation of a complete and functional EC layer on the inner surface of the scaffold. Numerous studies have demonstrated that the formation of fused monolayers of EC can be promoted to improve the patency of tissue-engineered vessels by seeding *in vitro* under shear stress [10,28,29]. In this study, We compared the differences in integrity and functionality of decellularised vascular implanted MSC after pulsed stimulation with increasing frequency and constant frequency and static culture at the same flow velocity. The aim is to achieve *in vitro* pulsed stimulation of the lumen with a single layer of fused endothelium that will function biologically when implanted in vivo, and to minimize the time to maturation of endothelialization for more favorable clinical applications.

Our results showed that static cultures showed a disordered arrangement of cells and more dead cells due to lack of nutrient renewal (Figure 2a), and after dynamic incubation, cells were arranged in the same direction of blood flow. The cells were significantly deformed, with maximum retention of cells stimulated by pulses at 60s frequency and gradually increasing frequency (Figure 2b, d). only a few cells remained in the 1s group, exposure to excessively high frequency pulse stimulation leads to cell detachment or rupture (Figure 2c). This is consistent with the results of Li that EC under sufficiently high shear stress has a lower rate of DNA synthesis than under static culture conditions, and that pulsatile flow reduces the number of cells entering the cell cycle. Pulsatile flow protects cells from apoptosis by inhibiting exogenous oxygen radicals, oxidizing LDL and serum depletion [30]. Recent experiments show that laminar flow reduces the number of cells entering the cell cycle, with the majority of cells being arrested in the G0 or G1 phase [31].

Electron microscopy of the inner surface of the lumen showed that cells covered the surface of the material in all four groups, with only a layer of membrane visible in static culture and no obvious cell morphology (Figure 3a); in flow conditions, cells were seen in long strips with pavement-like changes. 1S conditions showed that most cells were washed away and only a few residual cells were visible. Shear stress promoted the adhesion of endothelial cells to ECM and increased EC-ECM interactions. Such enhanced EC–ECM interaction may also play a significant role in promoting EC migration under flow [32].

Rotation promoted a uniform distribution of endothelial cells in the tubular structure, but the 1S frequency group did not see the formation of a continuous smooth endothelial layer because the cells were flushed. The experimental group with increasing frequency formed a smooth endothelial layer on the surface of the tubular lumen in response to flow stimulation. The basement membrane covered the decellularised inner surface. Preservation of intact elastin fibers increases elasticity and compliance, which can maintain vasomotor tone and homesstasis [33].

ECs on the intravascular surface exist in a highly dynamic and complex mechanical environment where endothelial cells sense mechanical stimuli through cell-matrix adhesion, cell-cell junctions and integrate different stimuli through complex transduction mechanisms to deliver them to the cell interior, resulting in changes in cell morphology, function and gene expression [34]. The dynamic culture groups flow at the same rate and eventually reach a shear stress level of 10 dyne/cm2, which is typical mean shear stress that in vivo arterial endothelial cells are exposed to [35]. Shear stress up to 10 dyn/cm2 is considered a suitable promoter for endothelial expression in arteries [36]. Platelet endothelial cell adhesion molecule-1 (PECAM-1, CD31) is an intercellular adhesion protein that translates biomechanics into downstream biochemical signals in response to shear stress. VE-cadherin acts as an adapter and plays an important role in maintaining the integrity and permeability of endothelial cell junctions, The transmembrane structural domain of VEGFR2 binds and VEGFR2 expression is increased, while also modulating the sensitivity of the shear stress sensor PECAM-1/VE-Cadherin. VE-cadherin, along with VEGFR2 and CD31, forms a key mechanosensory complex at EC junctions responsible for flow sensing. In the static culture group, none of the MSCs were expressed under stimulation without shear stress [Figure 5 A, E, H]. Under shear stress, CD31 expression was visible in all dynamic groups. 60S group and progressively increasing frequency group could intermittently shear stress modulated the distribution of regulated VE-cad along cell junctions, showing intermittent staining of VE-cadherin with more protein expression. 1S group was only visible in scattered cells due to rapid pulses. Dynamic culture groups all showed selective migration of MSC in the flow direction experimental groups maintained maximum cell integrity and protein expression with cells aligned along the flow direction. This is consistent with recent reports that the potential for MSC differentiation to endothelial cells on a decellularized vascular stroma was promoted by combining of physical-mechanical stimuli and biochemical factors [37,38].

Fibrous actin (F-actin) is an essential component of the cytoskeleton, providing mechanical support to cells and enabling rapid assembly and disassembly of the actin network to enable cell migration and adhesion. Under static culture conditions, MSC expressed only a small and randomly distributed amount of F-actin, and only scattered cells were seen in the 1S group with noticeable long changes. In both the constant 60S group and the gradually increasing frequency group, an increase of F-actin was observed around the nucleus, with the latter being thicker, denser, neatly arranged, and extended in the flow direction. It was shown that mechanical coupling of the apical membrane of unsheared endothelial cells to the cytoskeleton in which deformation at the surface was resisted primarily by F-actin, close interactions between the cytoskeleton and the cell membrane play a key role in cell shape rearrangement during flow [39]. Numerous studies have confirmed that under shear stress, EC enhances extracellular matrix secretion and increases the number of F-actin stress fibers to promote cell adhesion to the material surface and improves the mechanical reinforcement ability [40,41]. Also, after prolonged exposure to shear stress, cells overcome the limitations of cell-cell adhesion. Meanwhile, the cytoskeleton directly pulls on the nucleus, deforming the nuclear envelope. The resulting ellipsoidal shape and spatial rearrangement of cells reduce shear stress by 50%, thus minimizing intracellular stress [29].

Fibronectin (FN) is an extracellular matrix glycoprotein that acts as an adhesion molecule, anchoring cells to the extracellular matrix by mechanically coupling the actin cytoskeleton to the ECM via an adhesion complex synthesized by integrins, and Gong *et al*. showed that under physiological pulsatile flow conditions, the FN network is highly cross-linked and becomes thicker and denser [13]. Their frequency is 60S in one pulse, and the present experiment at 60S frequency similarly confirmed that FN is denser at 60s frequency than in static culture, while in the group of gradually increasing frequency, FN secretion is denser, and in the constant 1S group, cells are unable to tolerate leading to disruption of the FN network. FN matrix assembly is a cell-mediated process that affects cell growth, cell differentiation, and intercellular interactions, further facilitate the angiogenic cascade [42]. Only *in vitro* promotes cellular secretion of sufficient amounts of FN to resist natural shear stress after implantation *in vivo* [42,43].

Shear stress stimulates endothelial cells (ECs) through the activation of mechanosensory and integrins, tyrosine kinase receptors (TKRs), G proteins and G-protein – coupled receptors (GPCRs), ion channels, membrane lipids, and glycocalyx. Multiple signaling pathways coordinate to form mechanoresponsive networks to modulate endothelial cell (EC) phenotype and function [9,44]. Thrombomodulin, a glycoprotein expressed on the EC surface, not only prevents thrombin from causing fibrinogen coagulation and platelet aggregation but also activates protein C, which inactivates blood clotting factors [45]. Shear stress increases the expression of thrombomodulin at both the protein and gene levels in ECs (Figure 7d). By exposing porcine aortic endothelial cells to sinusoidal waveforms at three different frequencies, Heather found that at 1 Hz, several inflammatory transcripts were repressed relative to the steady stream, including IL-8 and VCAM [46].

During angiogenesis, endothelial cells are exposed to mechanical tension generated by matrix substrate, fluid shear stress, actin contractility and cell-cell junctional tension. Tension receptors at the junction, vinculin expression, strengthen the VE-cadherin connection to the actin cytoskeleton, thereby regulating adhesion between adjacent cells and allowing endothelial cells to migrate and rearrange themselves. thereby maintaining the integrity of the vasculature [47]. High expression at cell junctions was seen in the increasing frequency experimental group (Figure 7h). Vinculin represents a marker of vascular neogenesis.

In addition, shear stress promotes the release of vasodilators such as nitric oxide and prostacyclin from endothelial cells, which in combination with tissue plasminogen activator secretion helps to maintain graft patency and modulates different SMC phenotypes and inhibits excessive proliferative responses [48]. Bilodeau *et al*. kept endothelial cells at variable physiological frequencies of pulsatile blood flow and showed a more functional transcriptional profile, lower metabolic activity, expression of a more quiescent anti-inflammatory and anti-thrombotic phenotype, and higher nitric oxide production compared to a constant frequency [26].By reviewing cardiovascular physiology during embryonic and fetal development, the development of the heart and vascular system was promoted under conditions of low oxygen [49], less than 5% radial strain and crescendo heart rate [50]. In this study, MSC were implanted onto the surface of decellularized blood vessels and under pulsed stimulation with gradually increasing frequency, maximum cell retention was achieved and stem cells differentiated toward endothelial cells, forming a fused endothelial layer that is expected to function as an anti-thrombotic and inhibitor of endothelial proliferation after implantation, enabling individualized patient-specific therapy.

There are still some limitations in this experiment, we only characterized the vessels and cells after in vitro culture and did not perform in vivo validation in animal experiments to verify our findings. We will conduct fluorescent labeling of the implanted cells in the next step to investigate whether the cells implanted in vitro can tolerate the washout of real blood flow and to observe whether the implanted vessels can inhibit thrombosis and neointimal hyperplasia.

## 5. Conclusions

The decellularized vessels preserve the vasculature’s three-dimensional structure and have a surface topography suitable for MSC growth as well as good mechanical properties. The endothelialization of bone marrow mesenchymal stem cells on the lumen of the decellularized vasculature is enhanced by increasing the frequency of pulsed stimulation. After implantation, it is expected to have anti-thrombotic and anti-neointimal hyperplasia characteristics, ultimately improving the patency of small diameter TEVG.

## Abbreviation

endothelial cell (EC); mesenchymal stem cells (MSC); tissue-engineered vascular graft (TEVG); phosphate buffered saline (PBS); Immunofluorescence (IF);Extracellular matrix (ECM);Fibronectin (FN)
